The article "The Application of the GP Model to Manage Controllable Risk Factors in Stroke Patients with Diabetes Can Effectively Improve the Prognosis and Reduce the Recurrence Rate" was retracted in 2023. Reasons: signs of a paper mill; suspected computer-generated content; unreliable results or conclusions; concerns about the data.

# The Application of the GP Model to Manage Controllable Risk Factors in Stroke Patients with Diabetes Can Effectively Improve the Prognosis and Reduce the Recurrence Rate

**DOI:** 10.1155/2022/5413985

**Published:** 2022-08-05

**Authors:** Zhehua Zou, Kai Liu, Yunjing Li, Shuangyan Yi, Xiaotang Wang, Changying Yu, Haiying Zhu

**Affiliations:** ^1^Department of General Practice, The First Hospital of Qinhuangdao, Hebei 066000, China; ^2^Department of Neurology, Qinhuangdao Haigang Hospital, Hebei 066000, China; ^3^Department of Otorhinolaryngology Head and Neck Surgery, The First Hospital of Qinhuangdao, Hebei 066000, China

## Abstract

**Objective:**

The aim of this study is to examine the impacts of general practice model (GP) on prognosis and recurrence of stroke patients with diabetes.

**Methods:**

Ninety patients with stroke combined with diabetes mellitus admitted to our hospital from June 2019 to June 2020 were selected for the study and were randomly and equally divided into 45 cases each in the control and experimental groups for the prospective trial. The patients in the control group received routine treatment while those in the experimental group were treated with GP model. Comparison in treatment effects, patients satisfaction, psychological status, quality of life, glycosylated hemoglobin level, and stroke recurrence was carried out between the two groups.

**Results:**

The experimental group showed markedly better treatment effects (*P* < 0.05), higher satisfaction degree (*P* < 0.05), higher HAD (*P* < 0.05), GQOLI-74 score (*P* < 0.05), and BI index (*P* < 0.05), lower level of glycosylated hemoglobin (*P* < 0.05), and much lower recurrence rate (*P* < 0.05), as compared to the control group.

**Conclusion:**

The application of the GP model to manage controllable risk factors in stroke patients with diabetes can effectively improve the prognosis and reduce the recurrence rate, which is worthy of clinical application and promotion.

## 1. Introduction

Stroke is a common cerebrovascular disease often seen in the middle-aged and elderly population with a high incidence. Prompted by blocked blood circulation to the brain, stroke is among the diseases with extremely high mortality, together with heart disease and cancer. Globally, stroke mortality has declined, but the incidence of stroke and its sequelae have increased significantly over the past 30 years, with the global prevalence of diabetes estimated at 415 million adults in 2015 and diabetes care alone accounting for 12% of global health expenditure [1]. The incidence of stroke complicated by diabetes is 2∼3 times that of patients with stroke. The combination of stroke and diabetes mellitus is more complicated, which greatly affects the quality of life of patients and has a higher risk of disability or death.

In recent years, the incidence of stroke with diabetes has shown a rising trend due to unhealthy lifestyle brought by better material conditions, threatening life, and safety of the senior population [2–4]. Relevant studies have shown that the occurrence of stroke is highly relevant with hypertension, diabetes, atrial fibrillation, hypercholesterolemia, high salt diet, obesity, smoking, and drinking, among others. More than 75% of patients have different degrees of disability after stroke, which inflicts great pain and pressure to patients and their families. Diabetes mellitus is an independent risk factor for stroke. Long-term diabetes mellitus can cause vascular damage, leading to sclerosis of the cerebral arteries and narrowing of the vascular lumen, which is also an independent risk factor for cerebral infarction and haemorrhage [5]. Stroke includes both cerebral infarction and cerebral haemorrhage, which are clinically sudden in onset, but differ in that cerebral infarction is an ischaemic cerebrovascular disease that develops during sleep or in a quiet state. Cerebral haemorrhage occurs when the patient is agitated or active, and the patient's symptoms are characterised by a sudden onset of neurological deficits [6]. Therefore, effective treatment is required to drive down the recurrence rate. Since the reform and opening up, China has seen great progress in general practice. Stroke is one of the key chronic diseases in GP service [7–9].

The World Organization of Family Physicians defines a general practitioner as a person who provides comprehensive health care to every person who seeks it and, if necessary, arranges for other health professionals to provide related services [10]. Their role is not limited to the healing of the patient's organs, but to treat, care for, and counsel the patient in a variety of ways, including physical, psychological and social factors. The role of the general practitioner varies from country to country and region to region. For example, in cities in developed countries, GPs focus on the treatment of chronic diseases, early detection and referral of critically ill patients, and prevention and immunisation; in rural areas of developed countries or in developing countries, GPs may be involved in emergency care, baby delivery, community hospital services, and some less complex surgical procedures [11, 12]. Unlike specialists who focus on the treatment and research of difficult diseases in large general or specialist hospitals, GPs generally practise in institutions that provide primary health care services, helping people to look after most minor and common illnesses and providing good prevention services [10–13]. It has three main features: first, it emphasises continuous, comprehensive and individualised care for patients; second, it emphasises early detection and management of illnesses and disease, prevention of disease and maintenance of health; and it emphasises the uninterrupted management and service of patients in community settings and the co-ordinated use of other resources from within and outside the community when necessary [14, 15].

The prognosis for diabetic patients who have a stroke is poor because strokes generally cause glycaemic stress but are also an independent risk factor for the prognosis of cerebrovascular disease [16]. Studies have shown that the mortality rate for diabetic stroke patients is more than three times that of patients without stroke [17]. This study will analyze the effects of the management of the GP model on the prognosis and recurrence of stroke with diabetes patients.

## 2. Information and Methodology

### 2.1. General Information

Ninety patients with stroke combined with diabetes mellitus admitted to our hospital from June 2019 to June 2020 were selected as the study subjects and were equally divided into control and experimental groups using the random number table method, with 45 cases in each group. The study was reviewed and approved by the medical ethics committee of our hospital, and all patients themselves and their families were informed and provided written informed consent, and the study was approved by the ethics committee (approval NO. 20190412).

Inclusion criteria were as follows: (1) those with good clinical data; (2) those with a significant history; (3) those diagnosed with stroke combined with diabetes mellitus; and (4) those with communication skills and clear consciousness.

Exclusion criteria were as follows: (1) those with acute infection or chronic infection; (2) those undergoing other experiments; (3) those with poor compliance; and (4) those with mental disorders.

### 2.2. Methodology

The control group received routine treatment. After admission, medical staff would arrange a ward for the patient and provide guidance to take medicine and make a reasonable diet, etc.

The experimental group adopted the GP model for treatment: (1) A general practice management team was set up to formulate tailored plans for patients, provide regular intervention services, and adjust the plan in accordance with the actual situations. (2) Psychological intervention was carried out for patients. Stroke patients were susceptible to negative emotions such as fear, anxiety due to long-term treatment. Such negative emotions would affect the treatment and even aggravate the condition. Therefore, psychological intervention were required to help patients alleviate those negative emotions, establish a good and healthy mentality, and build confidence in treatment [18]. (3) The medical workers would evaluate the medication situation of patients, adjust the medication dose according to actual conditions, and provide necessary self-care guidance for patients. (4) The patients were guided for rehabilitation training, including passive activity, balanced position training, standing and walking, and daily life training. (5) Patients' diet was intervened in accordance with actual situations, which would underscore balanced nutrition, reduce spicy, raw and cold food, and supplement due amount of protein and vitamins. (6) Medical staff would maintain communication with patients and meet the requirements for patients in time to establish a friendly relationship with patients. At the same time, appropriate encouragement and guidance were given so that patients could feel warm, be relieved from the psychological pressure and pain, and maintain happy and pleasant mood [19].

### 2.3. Indicators

Satisfaction of patients after nursing was surveyed with the Patient Clinical Satisfaction Questionnaire designed by this department. The total score of the scale is 100 points, and the higher score means higher satisfaction.

The Hospital Anxiety and Depression Scale (HAD) was used to assess the emotional state of patients before and after intervention, with a total score of 42 points. The higher the score was, the more serious the anxiety and depression was.

The quality of life before and after intervention was assessed with reference to the Generic Quality of Life Inventory-74 (GQOLI-74) [20]. The scale was rated from four aspects, i.e. psychological function, physical function, social function, and material life, with a total score of 100. A higher score indicated a better quality of life.

Patients' everyday living ability was assessed by the BI Index Assessment Scale [21], with a total score of 100. The higher score represented the better ability to live daily [22].

The higher score indicated better mental state of patients.

The glycated hemoglobin level was calculated according to the 2013 edition of guideline for prevention and treatment of type 2 diabetes in China. The target of glycosylated hemoglobin control was <7%, It was recorded before the intervention of Education (admission), after the education intervention (at discharge), and at the first visit (at the end of 3 months after discharge) (Table1).

Comparison on the recurrence of stroke 3 months, 6 months, 9 months, and 12 months after discharge was made between the two groups.

### 2.4. Statistical Processing

In this study, SPSS20.0 and GraphPad Prism 7 (GraphPad Software, San Diego, USA) were used to analyze the data. The research included count data and measurement data using *χ*^2^ test, *t* test, and normality test. When *P* < 0.05, the difference was statistically significant.

## 3. Results

### 3.1. Comparison of General Information

There was no significant difference in age, gender, BMI, smoking, drinking, and residence between the two groups (*P* > 0.05) as shown in Table 2.

### 3.2. Comparison of Nursing Satisfaction between the Two Groups

The experimental group had a satisfaction rate of 71.11% (32/45), a comparative satisfaction rate of 22.22% (10/45), an unsatisfactory rate of 6.67% (3/45), and an overall satisfaction rate of 93.33% (42/45); the control group had a satisfaction rate of 44.44% (20/45), a comparative satisfaction rate of 28.89% (13/45), an unsatisfactory rate of 26.67% (12/45), with an overall satisfaction rate of 73.33% (33/45). The nursing satisfaction degree of the experimental group was significantly higher than that of the control group (*P* < 0.05) as shown in Figure 1.

### 3.3. Comparison of HAD Scores between the Two Groups

The HAD scores of the patients in the experimental group before and after the intervention were (35.81 ± 3.25) and (5.36 ± 1.21), respectively. The pre- and post-intervention HAD scores of patients in the control group were (35.88 ± 3.22) and (13.29 ± 2.53), respectively. The experimental group showed strikingly lower HAD score than the control group (*P* < 0.05) as shown in Figure 2.

### 3.4. Comparison of GQOLI-74 Scores between the Two Groups

The GQOLI-74 scores of patients in the experimental group before and after intervention were (46.44 ± 7.88) and (82.33 ± 4.98), respectively. The GQOLI-74 scores of patients in the control group before and after intervention were (46.72 ± 7.43) and (61.25 ± 4.22), respectively. The experimental group had remarkably higher GQOLI-74 score than the control group (*P* < 0.05) as shown in Figure 3.

### 3.5. Comparison of Recurrence Rates within One Year after Follow-Up of Patients

There was no significant difference in the recurrence rate of stroke within six months after discharge between the two groups (*P* > 0.05). The stroke recurrence rate in the experimental group was sharply lower than that in the control group 9 months and 12 months after discharge (*P* < 0.05) as shown in Table 3.

### 3.6. Comparison of BI Index Scores between the Two Groups

The BI index scores of patients in the experimental group before and after intervention were (51.24 ± 2.34) and (88.25 ± 1.27), respectively. The BI index scores of patients in the control group before and after intervention were (50.89 ± 2.56) and (69.77 ± 1.25), respectively. The experimental group had a much higher BI index score than the control group (*P* < 0.05) as shown in Figure 4.

### 3.7. Comparison of Glycosylated Hemoglobin Level Scores between the Two Groups

The difference of glycosylated hemoglobin level between the 2 groups was statistically significant. The level of glycosylated hemoglobin in the experimental group was lower than that in the control group (*F* = 5.720, *P* < 0.05); the difference was statistically significant at different time points, and there was interaction between groups and time (*F* = 103.067, *P* < 0.001). Further analysis of the separate effect, the level of glycosylated blood red protein in the experimental group was lower than that in the control group at the time of discharge and at the end of 3 months after discharge (*P* < 0.05).

## 4. Discussion

China's medical environment has seen great improvement with the advances of medical technology. Specialist services can no longer live up to people's needs for health services. Aiming to meet people's health needs, the Chinese scholars and experts have explored to establish a sound and distinctive system of general practitioners. Through continuous practice and exploration, progress has been achieved in the building of general practitioners team in China. The specification requirements have gradually become mature, and the training of general practitioners has seen increasingly profound and wide-ranging trend [23–26]. The main characteristics of stroke in diabetic patients are as follows: first, it occurs mostly in middle-aged and elderly diabetic patients; second, most diabetic patients with stroke have substandard long-term glycaemic control; third, stroke in diabetic patients may lead to massive cerebral infarction; and finally, if a diabetic patient has a stroke, it may induce severe acute complications of diabetes such as diabetic ketoacidosis or hyperosmolar hyperglycaemic syndrome. Therefore, diabetic patients need to have their blood glucose controlled and the risk of diabetes-related complications and cardiovascular disease assessed regularly and treated promptly and appropriately [16, 17].

GP diagnosis and treatment mode, an emerging medical pattern, serves stroke patients with a whole general practitioners team. It is mainly a family doctor mode constructed between general practitioners, patients and patients' families through the team service, in which doctors could have effective communication with patients, highly interactive and more convenient. It allows doctors to timely and accurately grasp the health information of patients and help them to recover better and faster [27–30]. Besides, GP treatment can improve patients' awareness of precaution. Through life guidance and psychological intervention, patients can maintain a positive mood, develop a good habit, and take a proactive part in receiving treatment, so as to help patients improve their quality of life. Stroke leads to a high mortality and disability rate, which not only poses a grave threat to the health and safety of patients, but also inflicts economic burden on patients, thus impeding the economic development and the stability of our society [31–34]. In the prevention and control of stroke, defensive management should be done in advance to eliminate the disease at its source, for which the general practitioner has an irreplaceable role to play in providing continuous and comprehensive healthcare services and medical treatment.

The results of this study have shown that the recurrence rate in the experimental group was significantly lower than that of the control group (*P* < 0.05), which was consistent with the research results of Caria et al [35]. who pointed out in the article that there was no significant difference in the recurrence rate of stroke within six months after the patient discharged from hospital (*P* > 0.05); while the recurrence rate of stroke registered 12.13% in the experimental group and control group 29.12% nine months after discharge (*P* < 0.05); the experimental group 13.74% and the control group 32.21% 12 months after discharge (*P* < 0.05), indicating a much lower recurrence rate of stroke in the experimental group than the control group (*P* < 0.05). Meanwhile, the level of glycosylated hemoglobin in the experimental group was lower than that in the control group, and the difference was statistically significant at different time points. It has been fully manifested that the GP model for the management of controllable risk factors can effectively reduce the recurrence rate of stroke, accelerate the rehabilitation process, and improve the quality of life for stroke patients.

Based on the risk of stroke in combination with diabetes mellitus, attention should be paid from prevention. Dialectical management in TCM can not only improve the overall state of the patient's body functions but also lower blood glucose, lower blood lipids, improve metabolism and protect blood vessels [36]. Because of the flexibility to treat each patient on an individual basis, dialectical management in TCM should be the first choice for stroke prevention and treatment. For patients with high risk factors for diabetes, or even those who already have mild abnormalities in blood glucose, lifestyle interventions and positive life modifications can be used to improve blood glucose [37]. Patients need to control their diet, combined with the medicated diet of traditional Chinese medicine. In addition to foods rich in cellulose and vitamins, some ingredients with nourishing yin and qi-enhancing effects can be added, including yam, etc. [36]. The application of the GP model in the management of controllable risk factors in nondiabetic stroke patients can effectively improve the prognosis and reduce the recurrence rate [38]. Therefore, in general, it has far-reaching clinical significance to incorporate traditional Chinese medicine methods into the GP model for promotion.

In summary, the controllable risk factors under the management of GP model can effectively drive down the recurrence rate and improve the prognosis of patients, which is worthy of further application and promotion in clinical practice. However, our trial sample size was small and of short duration, and recovery and daily monitoring of stroke combined with diabetes is a long-term process. We will need to follow-up with regular visits and expand the study to ensure clinical feasibility and widespread replication.

## Figures and Tables

**Figure 1:** Comparison of satisfaction between the two groups (*n* (%)). (a) shows the expression of nursing effect in the experimental group and (b) represents the expression of nursing effect in the control group. In the experimental group, the satisfaction rate was 71.11% (32/45), the more satisfied rate was 22.22% (10/45), and the dissatisfied rate was 6.67% (3/45). The total satisfaction rate was 93.33% (42/45). In the control group, the satisfaction rate was 44.44% (20/45), the more satisfied rate was 28.89% (13/45), and the dissatisfied rate was 26.67% (12/45). The total satisfaction rate was 73.33% (33/45). After nursing, there was a significant difference between the two groups (*x*^2^ = 6.480, *P*=0.011).

**Figure 2:** Comparison of HAD scores between the two groups (*x* ± *s*). The HAD scores of patients in the experimental group before and after intervention were (35.81 ± 3.25) and (5.36 ± 1.21), respectively. The HAD scores of patients in the control group before and after intervention were (35.88 ± 3.22) and (13.29 ± 2.53), respectively. ^*∗*^indicates a significant difference in HAD scores of patients in the experimental group before and after intervention (*t* = 58.901, *P* ≤ 0.001); ^*∗∗*^indicates a significant difference in HAD scores of patients in the control group before and after intervention (*t* = 37.005, *P* ≤ 0.001); ^*∗∗∗*^indicates a significant difference in post-intervention HAD scores between the two groups (*t* = 18.968, *P* ≤ 0.001).

**Figure 3:** Comparison of GQOLI-74 scores between the two groups ($\bar{X}$ ± *s*). The GQOLI-74 scores of patients in the experimental group before and after intervention were (46.44 ± 7.88) and (82.33 ± 4.98), respectively. The GQOLI-74 scores of patients in the control group before and after intervention were (46.72 ± 7.43) and (61.25 ± 4.22), respectively. ^*∗*^indicates a significant difference in GQOLI-74 scores in the experimental group before and after intervention (*t* = 25.828, *P* ≤ 0.001); ^*∗∗*^indicates a significant difference in GQOLI-74 scores in the control group before and after intervention (*t* = 11.407, *P* ≤ 0.001); ^*∗∗∗*^indicates a significant difference in GQOLI-74 scores between the two groups after intervention (*t* = 21.663, *P* ≤ 0.001).

**Figure 4:** Comparison of BI index scores between the two groups (*x* ± *s*). The BI index scores of patients in the experimental group before and after intervention were (51.24 ± 2.34) and (88.25 ± 1.27), respectively. The BI index scores of patients in the control group before and after intervention were (50.89 ± 2.56) and (69.77 ± 1.25), respectively. ^*∗*^indicates a significant difference in the BI index scores of patients in the experimental group before and after intervention (*t* = 93.250, *P* ≤ 0.001*);*^*∗∗*^indicates a significant difference in the BI index scores of patients in the control group before and after the intervention (*t = *44.456, *P* ≤ 0.001); ^*∗∗∗*^indicates a significant difference in BI index scores after intervention between the two groups (*t* = 69.568, *P* ≤ 0.001).

**Table 1:** Comparison of glycosylated hemoglobin levels between the two groups ($\bar{x}$ ± *s*, %).

Group	*n*	Before intervention	Discharge	3 months	Total	*F*	*P*
Experimental group	45	8.48 ± 0.96	6.01 ± 0.96	6.34 ± 0.99	6.58 ± 0.67	75.34	＜0.001
Control group	45	8.73 ± 1.07	6.55 ± 1.25	7.02 ± 1.25	7.52 ± 2.54	50.28	＜0.001
Total		8.61 ± 1.02	6.35 ± 1.17	6.72 ± 1.20	7.20 ± 1.47	103.067	＜0.001
*F*		1.361	5.282	8.183	5.720		
*P*		0.247	0.023	0.005	0.019		

**Table 2:** Comparison of general information of patients between the two groups (*n* (%)).

	Experimental group (*n* = 45)	Control group (*n* = 45)	*χ * ^2^ or t	*P*
*Age*	46.75 ± 3.32	46.69 ± 3.29	0.086	0.932

*Gender*			0.178	0.673
Male	23 (51.11)	21 (46.67)		
Female	22 (48.89)	24 (53.33)		

*BMI (kg/m * ^*2*^ * ）*			1.119	0.266
*Smoke*	26.27 ± 1.59	25.89 ± 1.63	0.045	0.832
Yes	20 (44.44)	21 (46.67)		
No	25 (55.56)	24 (53.33)		

*Alcohol*			0.178	0.673
Yes	22 (48.89)	24 (53.33)		
No	23 (51.11)	21 (46.67)		

*Residence*			0.050	0.822
Urban	31 (68.89)	30 (66.67)		
Rural	14 (31.11)	15 (33.33)		

**Table 3:** Comparison of stroke recurrence rates between the two groups (*n* (%)).

Group	*n*	3 months	6 months	9 months	12 months
Experimental group	45	1 (2.22)	5 (11.11)	5 (11.11)	6 (13.33)
Control group	45	3 (6.67)	7 (15.56)	13 (28.89)	14 (31.11)
*χ * ^2^		1.047	0.385	4.444	4.114
*P*		0.306	0.535	0.035	0.043

## Data Availability

The datasets used during the present study are available from the corresponding author upon reasonable request.

## References

[1] Tun N. N., Arunagirinathan G., Munshi S. K., Pappachan J. M. (2017). Diabetes mellitus and stroke: a clinical update. *World Journal of Diabetes*.

[2] Heldner M. R., Li L., Lovett N. G., Kubiak M. M., Lyons S., Rothwell P. M. (2018). Long-term prognosis of patients with transient ischemic attack or stroke and symptomatic vascular disease in multiple arterial beds. *Stroke*.

[3] Cuadrado-Godia E., Benito B., Ois A. (2020). Ultra‐early continuous cardiac monitoring improves atrial fibrillation detection and prognosis of patients with cryptogenic stroke. *European Journal of Neurology*.

[4] (2020). Clinical prognosis of FLAIR hyperintense arteries in ischaemic stroke patients: a systematic review and meta-analysis. *Journal of Neurology Neurosurgery and Psychiatry*.

[5] Chen R., Ovbiagele B., Feng W. (2016). Diabetes and stroke: epidemiology, pathophysiology, pharmaceuticals and outcomes. *American Journal of the Medical Sciences*.

[6] Morgenstern L. B., Hemphill J. C., Anderson C. (2010). Guidelines for the management of spontaneous intracerebral hemorrhage: a guideline for healthcare professionals from the American Heart Association/American Stroke Association. *Stroke*.

[7] Chiarelli A. M., Croce P., Assenza G. (2020). Electroencephalography-derived prognosis of functional recovery in acute stroke through machine learning approaches. *International Journal of Neural Systems*.

[8] (2020). Outcomes of acute stroke patients requiring mechanical ventilation: study protocol for the SPICE multicenter prospective observational study. *Neurocritical Care*.

[9] Buoite Stella A., Gaio M., Furlanis G. (2020). Prevalence of hypohydration and its association with stroke severity and independence outcomes in acute ischemic stroke patients. *Journal of Clinical Neuroscience: Official Journal of the Neurosurgical Society of Australasia*.

[10] Bentzen B. G., Bridges-Webb C., Carmichael L. (1991). *The Role of the General Practitioner/family Physician in Health Care Systems: A Statement from WONCA*.

[11] Moore M. (2006). Opportunities and challenges for GPs in the developing world. *Australian Family Physician*.

[12] Fletcher E., Campbell J., Pitchforth E. (2020). Comparing international postgraduate training and healthcare context with the UK to streamline overseas GP recruitment: four case studies. *BJGP open*.

[13] Zhang H., Xiao Y., Zhao X., Tian Z., Zhang S. Y., Dong D. (2022). Physicians’ knowledge on specific rare diseases and its associated factors: a national cross-sectional study from China. *Orphanet Journal of Rare Diseases*.

[14] Mathers N., Jones N., Hannay D. (1995). Heartsink patients: a study of their general practitioners. *British Journal of General Practice: The Journal of the Royal College of General Practitioners*.

[15] Baker R. (1996). Characteristics of practices, general practitioners and patients related to levels of patients’ satisfaction with consultations. *British Journal of General Practice: The Journal of the Royal College of General Practitioners*.

[16] Ergul A., Kelly-Cobbs A., Abdalla M., C Fagan S. (2012). Cerebrovascular complications of diabetes: focus on stroke. Endocrine, metabolic & immune disorders-drug targets (formerly current drug targets-immune. *Endocrine & Metabolic Disorders)*.

[17] Otiniano M. E., Du X. L., Ottenbacher K., Markides K. S. (2003 May 1). The effect of diabetes combined with stroke on disability, self-rated health, and mortality in older Mexican Americans: results from the Hispanic EPESE. *Archives of Physical Medicine and Rehabilitation*.

[18] (2020). Assessment of the manifestations of atrial fibrillation in patients with acute cerebral stroke—a single-center study based on 998 patients. *Neurological Research: An Interdisciplinary Quarterly Journal*.

[19] (2020). The role of diabetes mellitus on the thrombus composition in patients with acute ischemic stroke. *Interventional Neuroradiology: Journal of Peritherapeutic Neuroradiology, Surgical Procedures and Related Neurosciences*.

[20] Chang W. L., Lee J. T., Li C. R., Davis A. H. T., Yang C. C., Chen Y. J. (2020). Effects of heart rate variability biofeedback in patients with acute ischemic stroke: a randomized controlled trial. *Biological Research For Nursing*.

[21] Liang J., Zhang Z. (2020). Higher peripheral blood MiR-488 level predicts poor prognosis of acute ischemic stroke. *Clinical Laboratory*.

[22] Wang P., Fan J., Yuan L., Nan Y., Nan S. (2020). Serum neurofilament light predicts severity and prognosis in patients with ischemic stroke. *Neurotoxicity Research*.

[23] General Pediatricians’ Performance of Accreditation Agency’s Recommended Procedures (2020). A complementary analysis using administrative data and the knowledge translation model. *Journal of Continuing Education in the Health Professions*.

[24] Mulder R., Sorensen D., Kautoke S., Jensen S. (2020). Part II: using an integrated case model for delivering mental health services in general practice for Pacific people. *Australasian Psychiatry*.

[25] Byrne G. (2020). How the good lives model can complement mentalization-based treatments for individuals who have offended with anti-social personality disorder and general forensic mental health needs: practice update. *International Journal of Offender Therapy and Comparative Criminology*.

[26] Xurui L., Hui G., Ning X., Jianguo L. (2020). Discussion on the general practice initial diagnosis model based on process thinking. *Open Journal of Internal Medicine*.

[27] Jackson N., Haxton E., Morrison K. (2018). Reflections on 50 Years of neuroscience nursing: the growth of stroke nursing. *Journal of Neuroscience Nursing: Journal of the American Association of Neuroscience Nurses*.

[28] Webb A., Paolucci M., Mazzucco S., Li L., Rothwell P. M. (2020). Confounding of cerebral blood flow velocity by blood pressure during breath holding or hyperventilation in transient ischemic attack or stroke. *Stroke*.

[29] Ran Y., Wang Y., Zhu M. (2020). Higher plaque burden of middle cerebral artery is associated with recurrent ischemic stroke. *Stroke*.

[30] Tranchida G. V., Van Heest A. (2020). Preferred options and evidence for upper limb surgery for spasticity in cerebral palsy, stroke, and brain injury. *Journal of Hand Surgery*.

[31] Dhar R., Chen Y., Hamzehloo A. (2020). Reduction in cerebrospinal fluid volume as an early quantitative biomarker of cerebral edema after ischemic stroke. *Stroke*.

[32] Mackay M. (2020). Focal cerebral arteriopathy and childhood stroke. *Current Opinion in Neurology*.

[33] Pavlova O. N., Abdurashitov A. S., Terskov A. V., Semyachkina-Glushkovskaya O. V., Pavlov A. N. (2020). Synchronization of cerebral and peripheral blood flow at the latent stage of stroke. *International Journal of Modern Physics C*.

[34] Gao B. Y., Sun C. C., Xia G. H. (2020). Paired associated magnetic stimulation promotes neural repair in the rat middle cerebral artery occlusion model of stroke. *Neural Regeneration Research*.

[35] Caria F., Zedde M., Gamba M. (2019). The clinical spectrum of reversible cerebral vasoconstriction syndrome: the Italian Project on Stroke at Young Age (IPSYS). *Cephalalgia*.

[36] Covington M. B. (2001). Traditional Chinese medicine in the treatment of diabetes. *Diabetes Spectrum*.

[37] Shrivastava S. R., Shrivastava P. S., Ramasamy J. (2013). Role of self-care in management of diabetes mellitus. *Journal of Diabetes and Metabolic Disorders*.

[38] Olsson T. M., Viitanen M., Asplund K., Eriksson S., Hägg E. (1990). Prognosis after stroke in diabetic patients. A controlled prospective study. *Diabetologia*.

